# Food for Thought: Machine Learning in Autism Spectrum Disorder Screening of Infants

**DOI:** 10.7759/cureus.18721

**Published:** 2021-10-12

**Authors:** Sohaib Siddiqui, Luxhman Gunaseelan, Roohab Shaikh, Ahmed Khan, Deepali Mankad, Muhammad A Hamid

**Affiliations:** 1 Department of Obstetrics and Gynaecology, Women’s College Hospital, Toronto, CAN; 2 Department of Pediatrics, Saba University School of Medicine, The Bottom, BES; 3 Department of Family Medicine, University of British Columbia, Vancouver, CAN; 4 Department of Pediatrics, Southern Health & Social Care NHS Trust, London, GBR; 5 Department of Developmental Pediatrics, University of Toronto, Toronto, CAN; 6 Department of Pediatrics, University of Toronto, Toronto, CAN

**Keywords:** autism spectrum disorder (asd), machine learning (ml), autistic behavior, screening, diagnosis

## Abstract

Diagnoses of autism spectrum disorders (ASD) are typically made after toddlerhood by examining behavioural patterns. Earlier identification of ASD enables earlier intervention and better outcomes. Machine learning provides a data-driven approach of diagnosing autism at an earlier age. This review aims to summarize recent studies and technologies utilizing machine learning based strategies to screen infants and children under the age of 18 months for ASD, and identify gaps that can be addressed in the future. We reviewed nine studies based on our search criteria, which includes primary studies and technologies conducted within the last 10 years that examine children with ASD or at high risk of ASD with a mean age of less than 18 months old. The studies must use machine learning analysis of behavioural features of ASD as major methodology. A total of nine studies were reviewed, of which the sensitivity ranges from 60.7% to 95.6%, the specificity ranges from 50% to 100%, and the accuracy ranges from 60.9% to 97.7%. Factors that contribute to the inconsistent findings include the varied presentation of ASD among patients and study design differences. Previous studies have shown moderate accuracy, sensitivity and specificity in the differentiation of ASD and non-ASD individuals under the age of 18 months. The application of machine learning and artificial intelligence in the screening of ASD in infants is still in its infancy, as observed by the granularity of data available for review. As such, much work needs to be done before the aforementioned technologies can be applied into clinical practice to facilitate early screening of ASD.

## Introduction and background

Autism spectrum disorder (ASD) is a complex neurodevelopmental disorder characterized by persistent deficits in social communication and social interaction across multiple contexts, as well as restricted repetitive patterns of behavior, interests or activities [1]. The prevalence of ASD has increased worldwide in recent years. The CDC released a report citing a prevalence of ASD of 16.8 per 1000 in 2014, a significant increase from 14.7 per 1000 in 2010 [2].

Currently, the American Academy of Pediatrics recommends that all children receive screening tests for ASD and language development, conducted at 18- and 24-month well-child visits [3]. Early detection and intervention will result in improved social functioning and better long-term outcomes [4]. Zuckerman et al. concluded that children who were diagnosed late were more likely to be treated with medications or alternative medication, whereas children diagnosed early responded well to conventional ASD therapy such as speech therapy, and monitoring by a pediatric psychiatrist [5].

When screening for ASD, pediatricians utilize screening tests to look for pathognomonic behavioural features, such as not babbling by the age of 12-15 months, being unable to speak words by age two, and inability to form basic sentences by age three [4].

There are multiple ASD screening tests to screen for autism under 24 months of age, such as the Modified Checklist for Autism in Toddler (M-CHAT) and the Screening Tool for Autism in Two-Year-Olds (STAT) [3]. These tests however have low sensitivity and positive predictive value (PPV) when used in children in this age group. Their performance also varies considerably by the cut off values used. The Modified Checklist for Autism in Toddlers (M-CHAT) is a popular two-stage screening tool to identify autism in infants. However, while it does have a PPV of 0.61 in those aged 24 to 30 months, the PPV drops to 0.28 when examining toddlers aged 16 to 23 months [3]. Autism is difficult to detect early in life as the social deficits and other core behavioral features are difficult to identify until the first birthday and may not peak until several months later [4], and behaviours in typically developing toddlers overlap with ASD deficits, such as repetitive behaviours and restricted interests. Screening tests such as the M-CHAT also vary in performance when administered in languages other than English. When assessing a Spanish translation of the M-CHAT in a community in Spain, Canal-Bedia et al. found a PPV of 0.19 [3].

As such, there exists an unmet need to develop a method of ASD screening targeting children by 18 months of age that is more reliable than the current screening tests without variances in performance due to language.

New technologies such as machine learning are promising tools to complement current clinical protocols. Machine learning describes how computers can learn patterns from empirical data. Artificial intelligence describes technologies that can perform cognitive functions, such as recognition of symptoms, classification, diagnosis, and prediction of outcomes based on data obtained through various means [6]. Machine learning is an aspect of artificial intelligence that allows a system to improve by ‘learning’ from an encounter. Current machine learning approaches include neural networks, decision trees, rule-based classifiers, and support vector machines [6]. By capturing data and making connections that aren’t apparent by human observation alone [6], how can these technologies be harnessed to improve screening methods for ASD in clinical practice?

We hope to explore this question by summarizing current efforts to incorporate machine learning technology in the screening of ASD in children less than the age of 18 months through various modalities such as epigenetic biomarkers, behavioural patterns, acoustic prosody, structural/functional MRI, EEG, and app-based platforms.

## Review

Methods

A literature review of studies using machine learning technology in the early screening of ASD was conducted on peer-reviewed primary journal articles listed in PubMed and Medline from the last 10 years (February 2011 to February 2021). The search terms used were (MRI OR EEG OR eye tracking OR prosody OR intonation OR intensity OR pitch OR speech rate OR voice quality OR acoustic OR movement OR AOSI OR MESL OR VABS) AND (autis* OR Asperger) AND (machine OR artificial intelligence) AND (Infant OR Toddler) Filters applied into PubMed included: Infant: birth-23 months. Studies were excluded if they were 1) methodological papers, 2) animal studies 3) reviews, meta-analyses or editorials. Based on these criteria, 65 papers were excluded. The remaining 23 articles underwent full text review and removed from analysis if: 1) mean age was more than five, 2) genetics or neuroimaging scans were used as the main source of data, 3) machine technology was not the major method employed in the study. Fourteen studies were excluded after full text review, leaving nine studies to be included in the analysis.

Results

We describe our findings by introducing how machine learning can be utilized to complement existing ASD assessment tools and new behavioral components, with the potential to improve early screening of ASD. Table 1 summarizes the studies that aim to screen for ASD in children less than 18 months.

**Table 1:** Summary of studies using machine learning technology in children <18 months old. ADOS: Autism Diagnostic Observational Schedule, ADTree: alternating decision tree, AOSI: Autism Observational Scale for Infants, ASD: autism spectrum disorder, AUC: area under the curve, DWI: Diffusion Weighted MRI, ECBQ: Early Childhood Behavior Questionnaire, eGeMAPS: (Geneva Minimalistic Acoustic Parameter Set), FcMRI: Functional Connectivity MRI, HR: high risk, IBQ-R: The Infant Behavior Questionnaire- Revised, LR: low risk, m: months, M-CHAT-R/F: Modified Checklist for Autism in Toddlers-Revised/Follow-Up,  mMSE: modified multiscale entropy, NPV: Negative Predictive Value, PPV: Positive Predictive Value, RF: random forest, SVC: support vector classification, SVM: support vector machine, TD: Typical development; VABS: Vineland Adaptable Behavior Scale, yrs: years

Author	Sample Size	Age at Screening	Data Type	Method	Accuracy
Santos et al. (2013) [7]	23(HR), 20 (LR)	18 m	Acoustic prosodic features	SVM, neural network	Accuracy (%): 79.1-97.7, AUC (%): 66-97, Sensitivity (%): 69.6-95.6, Specificity (%): 50-100
Pokorny et al. (2017) [8]	10(pre-ASD), 10 (TD)	10 m	Acoustic prosodic features	SVM, neural network	Accuracy (%): 75
Bussu et al. (2018) [9]	161 (HR), 71 (LR)	8.5m, 14.5 m	VABS, AOSI	SVM	Accuracy (%): 66.4 (8 m), 64.4 (14 m), Sensitivity (%): 68.8 (8m), 67.5 (14m), Specificity (%) 64.4 (8m) 67.5 (14m), AUC (%) 69.2 (8m), 70.8 (14m)
Pijl et al. (2019) [10]	170 (HR), 77 (LR)	14 m	Temperament: IBQ-R	SVM	Accuracy (%): 60.9, AUC (%): 64.4, Sensitivity (%): 69.6, Specificity (%): 59.2, PPV (%): 26.6, NPV (%): 90.3
Bahado-Singh et al (2019) [11]	14 (cases), 10 (controls)	1m	CpG Methylation sites	SVM	AUC (%): 100, Sensitivity (%): 97.5, Specificity (%): 100
Emerson et al (2017) [12]	59 (HR)	6m	FcMRI: Functional brain connections	SVM	PPV (%): 100, NPV (%): 96, Sensitivity (%): 81.8
Jin et al. (2015) [13]	40 (HR), 40 (LR)	6m	DWI: White matter tract abnormalities	SVM	Accuracy (%): 76, AUC (%): 80.3, Sensitivity (%): 72, Specificity (%): 79.3, PPV (%): 78.7, NPV (%): 75.5
Bosl et al. (2011) [14]	46 (HR), 33 (TD)	6-24 m	Resting State EEG data	mMSE	Accuracy (males) (%): 100 (9m), 70-90 (12-18m)
Miron et al (2015) [15]	30 (1-3m), 40 (12-42m)	1-3m, 12-42m	Auditory brainstem EEG responses	SVM	Sensitivity (%): 70, Specificity (%): 80

Acoustic Prosody

Many infants with ASD manifest with unique acoustic features of their babbling and speech during infancy. Santos et al. (2013) attempted to use this difference in acoustic features between ASD and typically developing (TD) infants as indicators for classification [7]. Acoustic prosodic features of babbles and cries of 18-month toddlers were extracted and used to train support vector machine (SVM) and probabilistic neural networks, allowing for classification accuracy up to 97.7%. Pokorny et al. (2017) analyzed vocalisations from parent-child interaction recordings on the eGeMAPS acoustic features set used for clinical speech analysis applications [8]. This allowed for differentiation between vocalisations of infants later diagnosed with ASD and controls. This process was automated by linear kernel support vector machines and a short-term memory neural network, achieving an accuracy of 75% for identifying pre-ASD subjects.

Behavioural Features

Infants with ASD also manifest with unique behavioural features, much of which can be documented and analyzed through a variety of surveys completed by the child’s parents. Bussu et al. (2018) used support vector machine (SVM) algorithms to screen 14-month-old infants for behavioural patterns that would help diagnose ASD using developmental evaluations such as the Mullen Scales of Early Learning (MSEL) and Vineland Adaptable Behavior Scale (VABS) [9]. Compared to the clinical judgments made by researchers using Autism Diagnostic Observation Schedule (ADOS) and Autism Diagnostic Interview Revised (ADI-R), the machine learning based approach was able to successfully screen infants at 14 months of age, who would later be diagnosed with ASD at three years of age, with an accuracy of 64.4%.

Pijl et al. (2019) used support vector machine (SVM) algorithms with effortful control to screen infants for differences in parent-reported temperament for high-risk and low-risk siblings at eight, 14, and 24 months, with diagnosis taking place at age three [10]. To assess for temperament in eight- and 14-month-old infants, the Infant Behavior Questionnaire-Revised (IBQ-R) scale was used. Study results reveal that high risk siblings who eventually go on to be diagnosed with ASD could not be identified accurately, with a PPV of 26.6% using data obtained at 14 months of age, whereas high risk infants who did not get diagnosed with ASD could be accurately identified, with an NPV of 90.3%.

Epigenetic Markers

Epigenetic factors may play a significant role in ASD development [16]. Epigenetics involve alterations in gene function not due to mutations, such as environmental factors. Bahado-Singh et al. (2019) used deep learning and ingenuity pathway analysis (IPA) to examine leukocyte epigenomic markers linked to development of ASD, as a screening tool for newborn infants [11]. These genes (MECP2, EIF4E, FYN, SHANK1, VIM, LMX1B, GABRB1, SHDAP3 and PACS2) are among the 249 genes found to have significant dysregulated CpG methylation, a finding strongly correlated with ASD development. Identifying significant CpG sites within these genes and determine whether they were hypomethylated or hypermethylated, and the use of deep learning was used to screen for ASD in newborns, with 97.5% sensitivity and 100.0% specificity, with an area under the curve (AUC) (95% CI) of 1.0 [11].

MRI Studies

MRI studies (Diffusion MRI, Structural MRI, Functional MRI) may be used along with machine learning to screen individuals for ASD in patients as young as neonates [17].

Functional MRI (FcMRI) links functional organization of the human brain to individual cognitive profiles, and when coupled with machine learning, can predict brain maturation and the possible development of ASD [12]. Emerson et al. (2017) performed prospective neuroimaging of 59 six-month-old infants with a family history of ASD, identifying functional brain connections with support vector machine (SVM) models that correlated with 24-month clinical assessment scores of ASD features, such as social behavior, language, motor development, and repetitive behavior [12]. This screening method had a PPV of 100%, and sensitivity of 81.8%, and negative predictive value of 96%, correctly predicting nine out of 11 infants at six months who were diagnosed with ASD at 24 months.

Diffusion‐weighted MRI (DWI) is a powerful non-invasive neuroimaging technique that assesses white matter (WM) integrity and connectivity [18]. DWI has been used to study white matter pathways of neurological conditions including ASD [19]. White matter tract abnormalities were ahead of ASD symptom manifestations in the first year of life. For example, the failure of orienting gaze and visual attention implied abnormal development of posterior cortical circuits in seven-month-old ASD infants [20]. Jin et al. (2015) performed prospective neuroimaging of 40 high risk and 40 low risk six-month-old infants with a family history of ASD, identifying white matter tracts through diffusion MRI with multikernal support vector machine (SVM) models that correlated with a diagnosis of ASD at 24 months [13]. This screening method achieves an accuracy of 76%, sensitivity of 72%, specificity of 79.3%, PPV of 78.7%, NPV of 75.5%, and AUC of 80.3%.

EEG Studies

Electroencephalography (EEG) utilizes scalp electrodes to analyze brain electrical activity to assess for neurological diseases. ASD is characterised by a decrease in synchronization between EEG electrodes when using coarse-grained entropy. EEG may therefore be able to screen for ASD [14]. Bosl et al. (2011) was able to effectively screen children aged six to 24 months for ASD by using a modified multiscale entropy (mMSE) of resting state EEG data. In males, classification accuracy was close to 100% at nine months and remained high (70% to 90%) at ages 12 and 18 months. In females, classification accuracy was highest at age six months, but declined afterwards [14]. Miron et al. (2015) investigated auditory brainstem response (ABR) as a valid marker for ASD risk [15]. Prolonged ABR latency has been associated with ASD in children. In this study, 30 infants up to age six months were assessed for ABR latency, and later was followed up with ASD assessment at toddlerhood. Classification of infants who later developed ASD and case‐matched controls using this measure enabled accurate identification of ASD infants with 80% specificity and 70% sensitivity.

Discussion

The purpose of this literature review was to identify studies aiming to develop applied machine learning technologies to screen for ASD in children less than 18 months old. A total of nine articles were reviewed that used machine learning methods to screen for ASD in infants (Table 1). Two articles reviewed used behavioural screening tests such as VABS, AOSI, and IBQ-R, with support vector machine as the analysis method. With accuracy ranging from 60.9% to 66.4%, these studies were not able to make reliable classification or prediction of ASD development in participants under 18 months. Sensitivities ranging from 68.8 to 69.6% and specificities from 59.2% to 67.5%, suggests possible over referral in both high risk and normal risk infants.

Studies that used acoustic features to screen for ASD were more seemingly more successful than those utilizing rating scales, as witnessed by the increased accuracy ranging from 79.1-100%. The sample size of the behavioural scales group was much larger than the acoustic prosodic features group, which may reflect the increased availability and ease of data collection from parental questionnaires as opposed to primary acoustic data. Studies that rely on questionnaires answered by parents, however, can introduce an element of human error, something which is not seen in studies relying on acoustic features. Developing machine learning-based screening tools that rely on primary data such as acoustic features, eye tracking, and movement abnormalities will allow for screening utility for all infants, irrespective of parental knowledge of ASD.

A study investigating epigenetic markers that are associated with ASD (CpG methylation sites) was very effective in predicting development of ASD in infants less than 18 months, as seen with the sensitivity and specificity of 97.5% and 100% respectively [12]. Further studies examining these markers need to be conducted, but this shows that screening tests relying on epigenetic markers do have potential in screening for ASD. With this technology, infants can be screened for ASD remotely by submitting a buccal swab DNA sample for laboratory testing. Alternatively, this screening can be performed as part of routine neonatal screening testing. 

MRI-based screening tests were investigated in several studies, evaluating either functional brain connections [14] or white matter tract abnormalities [13]. MRI-based screening modalities for ASD are more accurate than behavioural screening tests, with accuracy of 76% and sensitivity and PPV ranging from 72-81.8% and 78.7-100% respectively. Unlike epigenetic, acoustic or behavioural screening tests, however, MRI-based screening tests require access to MRI-capable facilities, and thus may not be viable for widespread ASD screening, especially in remote regions.

EEG data measuring resting state and auditory brainstem responses were evaluated, both revealing better accuracy, sensitivity and specificity in screening for ASD compared to behavioural studies. Bosl et al. (2011) investigated resting state EEG data as a screening modality for ASD, and found that accuracy was best when infant was male and nine months old, at 100%, and declined in female gender, or as the infant got older. The developmental differences as a result of gender can be explained by a familial endophenotype that expresses autism in males longer than females [14]. Miron et al. (2015) examined auditory brainstem responses in infants under 18 months and obtained a sensitivity and specificity of 70% and 80% respectively. Like MRI screening tests, EEG-based screening tests require access to EEG-capable facilities, and thus may not be viable for widespread and remote ASD screening.

Numerous studies currently exist that examines the efficacy of machine-based learning in screening and diagnosis of ASD in older children, with significant sensitivity, specificity and accuracy. These studies utilize parameters such as eye tracking fixation times [19], hand coordination [20] and video analysis of upper limb movements [13]. While these studies only support the application of machine learning in the screening of ASD in children who are past infancy, they reveal potential parameters that can be used in screening infants, and is therefore a target for further research.

Current Screening Technologies

The benefits of a machine learning-based tool for the early screening of ASD are numerous. As previously mentioned, early interventions can improve ASD clinical outcomes. Also, through machine learning-based technologies, databases can be developed that provide a larger sample of a child’s speech compared to a traditional exam conducted at a physician’s office, which relies heavily on the memory of parents and the assessment itself is a few minutes resulting in the sample not being as accurate and relatively small.

Several projects are currently underway that aim to develop an ASD screening modality that is portable and utilizes machine learning technology (Table 2).

**Table 2:** Summary of applications using used to detect autism spectrum disorders and developmental delay in children <18 months old.

App Name	Organization(s)	Screening Parameters
Sense to Know	Duke University	Video capture of child behaviour and response to video/game-based stimuli Gaze, affect, head pose, and facial landmark dynamics
Cognoa	Stanford University, Harvard University	Video led assessment: parents watch videos to identify specific patterns associated with autism, before examining their children and completing a survey via. Mobile app. Features examined: Making consistent eye contact with others, showing toys to others, engaging in pretend play, directing other people’s attention by pointing, responding when name is called, using gestures such as waving goodbye, copying or imitating other people’s actions.
EarlySee	University at Buffalo	Gaze detection and facial expression in order to detect the risk of autism The app will display multiple images and videos and track the eye movements of the child while the video is played.

Sense to Know is an early autism screening app developed by Duke University [21]. The app presents research-based stimuli that elicit behaviors related to ASD in children from 12-30 months. While the child enjoys a video or game in an unconstrained setting, the front camera of the device is used to capture their reaction and behavior. Computer vision and AI tools allow the researchers to screen for behaviors elicited from the videos related to autism, including gaze, affect, head pose, and facial landmark dynamics to screen for autism. The goal is to produce scalable, accessible, and universal access to the best screening tools available to these children and their families.

Cognoa is an early autism screening app developed by Stanford and Harvard Medical School [22]. Parents are asked to input data of their child by questionnaires about their typical behaviors and uploading short videos. Using machine learning, the app can analyze and predict if a child is at risk for developmental delay or autism. It can help identify red flags in development but also help with analyzing progress on normal development. They have a data set of 10,000 families with varying degrees of developmental delay and or autism spectrum disorder. System is currently 80-94% accurate. The app will generate reports that parents to take to clinicians for further evaluation.

EarlySee is another autism screening app currently being developed by the University at Buffalo [23]. The app utilizes gaze detection and facial expression in order to detect the risk of autism. The app will display multiple images and videos and track the eye movements of the child while the video is played. Typically, the normal reaction is to focus on people’s faces and eyes to be able to detect any abnormalities. If a child is not making appropriate eye contact then it should be a red flag for a parent. This app can potentially help identify children earlier for potential signs and symptoms.

Many of these projects involve applications installed onto portable devices that would allow children to be tested in their own home environment as opposed to an outpatient clinic which can reduce the incidence of confounding variables. In this environment, children are more likely to display their baseline and natural behaviour which will allow for their level of functioning to be established on a more accurate basis. This technology could also help stratify children who are at high risk for ASD and warrant further diagnosis.

Certain precautions need to be adhered to when utilizing machine-based learning tools for the early screening of ASD. As with any personal data, especially in the health care sector, privacy is paramount. Any technology that interacts with patients should adhere to the most stringent privacy and data protection laws. Parents should be in control of when and how their child’s data is collected, and any voice and video data should not be stored, but instead analyzed for the sole purpose of increasing the strength of the algorithm.

Another potential limitation of such technology is the inherent bias that may be introduced into the algorithm. Algorithms can be biased based on the type of data that is initially inputted. If a particular data set is not diverse, it may compound certain biases. One way to remedy this issue is to collect a large set of training data that is continually growing and accounts for a diverse infant population who are both developmentally normal and delayed. This is particularly relevant when it comes to speech as multilingual children with different speech patterns may otherwise be screened as developmentally delay. 

## Conclusions

New technologies such as artificial intelligence and machine learning are promising tools for the early screening of ASD. The paucity of available studies that examine machine learning technologies in infants less than 18 months of age is a significant limitation of this literature review. Future studies should be directed towards identifying behavioural biomarkers associated with ASD in infants. This can help develop machine learning-based ASD screening tools for infants that are viable in clinical practice. These solutions can potentially lead to earlier interventions and improved clinical outcomes.
